This article has been retracted.

# hMSCs Migrate under the Chemotaxis of CXCL-13 and Enhance Islet B Cell Activity through p-AKT Signaling Pathway in High-Glucose Environment

**DOI:** 10.1155/2022/5430175

**Published:** 2022-01-07

**Authors:** Yongtao Li, Wenshan Bian, Yang Jiang, Danyang Liu, Lei Shen

**Affiliations:** ^1^Department of Anatomy, Basic Medical College, Qiqihar Medical University, Qiqihar 161006, Heilongjiang, China; ^2^Department of Histology and Embryolog, Basic Medical College, Qiqihar Medical University, Qiqihar 161006, Heilongjiang, China

## Abstract

As a common clinical chronic disease, the incidence of diabetes is increasing year by year. According to the latest statistics from the International Diabetes Federation, as of 2019, the global prevalence of diabetes has reached 8.3%. This study aims to investigate the effect of CXCL-13 on the migration ability of human mesenchymal stem cells (hMSCs) and to clarify the specific molecular mechanism of the protective effect of hMSCs on islet B cells. The hMSCs were cultured in high-glucose environment, and the effect of CXCL-13 on the migration ability of hMSCs was determined by Transwell experiment. After coculture of hMSCs and islet B cells, the activity of cells was detected by CCK8 assay, the expression of Ki-67 in cells was detected by RT-PCR, and the expression of P53 was detected by Western blot to investigate the effect of hMSCs on the proliferation and apoptosis of islet B cells. The effect of hMSCs on the function of islet B cells was determined by glucose stimulated insulin secretion experiment. Transwell experiment results showed that CXCL-13 could promote the migration of hMSCs to islet B cells in high-glucose environment. The results of CCK-8 showed that the cell activity in the coculture group was significantly higher than that of the other groups, and RT-PCR showed that the expression of Ki-67 was significantly increased in the coculture group of hMSCs and islet B cells. The results of Western blot showed that the expression of P53 was significantly decreased in the coculture group, and the glucose stimulated insulin secretion test showed that insulin secretion was significantly increased. It was found that after the inhibition of ATK, cell activity was significantly reduced, and apoptosis was significantly increased. Meanwhile, the expression of Ki-67 was inhibited, the expression of P-53 was significantly increased, and insulin secretion was significantly reduced. To sum up, in a high-glucose environment, CXCL-13 effectively promoted the migration of hMSCs, and hMSCs protected the activity and function of islet B cells through Akt signaling pathway.

## 1. Introduction

In 2019, the number of diabetic patients in China has reached 116 million, the largest diabetic patient number in the world, and about 90% of them are type 2 diabetes patients [1]. The mechanism of the development of type 2 diabetes is that long-term chronic hyperglycemia significantly inhibits the activity of islet B cells and promotes the apoptosis of islet B cells [2, 3]. The decrease in islet B cells number leads to decreased function of islet B cells [4]. Therefore, the effective protection of the activity of islet B cells in high-glucose environment has become a new target for the treatment of type 2 diabetes. [5]

As seed cells, stem cells are expected to be used in the treatment of a variety of diseases due to their self-renewal and multidirectional differentiation abilities [6]. Previous studies have also shown that mesenchymal stem cells could secrete a variety of growth factors and extracellular matrix and had significant regulatory effects on angiogenesis, immune, and inflammatory responses [7]. Therefore, mesenchymal stem cells are expected to be an adequate tool in the effective treatment of type 2 diabetes. Jiang [8] injected placenta-derived mesenchymal stem cells into patients and recorded the follow-up observations after injection. The results showed that 6 months later, the demand for insulin and the level of glycosylated hemoglobin were significantly reduced in the group injected with stem cells. Liu et al. [9] injected mesenchymal stem cells into patients with type 2 diabetes and found that fasting blood glucose was significantly reduced after stem cell inhibition. These studies also proved that mesenchymal stem cells have good effect on the treatment of type 2 diabetes. Studies have shown that high-glucose environment could inhibit the expression of Ki67 in cells. As a protein related to cell proliferation, the inhibition of Ki67 also proves that high-glucose environment may have a certain negative effect on cell proliferation [10]. Previous studies have also shown that mesenchymal stem cells could significantly inhibit the expression of P53 in fibroblasts in high-glucose environment. As a protein related to cell aging, the inhibition of P53 expression also proved that stem cells could inhibit cell aging in high-glucose environment [11, 12]. These studies also suggested that stem cells could promote the proliferation of B cells and inhibit their senescence. However, there are still some deficiencies in the treatment of type 2 diabetes with mesenchymal stem cells. For stem cell treatment, it still requires great efforts to explore the way to effectively aggregate mesenchymal stem cells in target organs and target cells after injection [13]. At the same time, there is no consensus on the specific molecular mechanism of mesenchymal stem cells in the treatment of type 2 diabetes. In order to increase the local aggregation efficiency of mesenchymal stem cells and enhance their migration ability, researchers attempted to promote the local aggregation and migration of mesenchymal stem cells with local addition of chemokines (CXCL) [14]. Yi et al. [15] loaded CXCL-13 into hydroxyapatite microsphere and found that CXCL-13 could significantly improve the migration rate and efficiency of mesenchymal stem cells. However, no studies have reported the role of CXCL-13 in promoting the immigration of mesenchymal stem cells into islet B cells. Previous studies have also shown that the protein kinase (AKT) signaling pathway is one of the major signaling pathways that protect the function and activity of islet B cells [16], and it plays an important role in the function and survival of islet cells. However, no studies have reported whether mesenchymal stem cells can protect islet injury in high-glucose environment through AKT signaling pathway.

In this study, mesenchymal stem cells and islet B cells were cultured in a high-glucose environment, and CXCL-13 was added into the culture medium to clarify the effect of CXCL-13 on the migration ability of mesenchymal stem cells in a high-glucose environment. The specific mechanism of the protective effect of mesenchymal stem cells on islet B cells was explored by adding AKT pathway inhibitors into the culture medium. The results of our study showed that CXCL-13 could effectively promote the migration and aggregation of hMSCs to islet B cells in high-glucose culture environment. At the same time, hMSCs could protect the activity of islet B cells through the AKT signaling pathway, promote the proliferation of islet B cells, and inhibit the apoptosis of islet B cells in the same environment.

## 2. Experimental Methods

### 2.1. Cell Lines and Cell Culture

Human mesenchymal stem cells and human islet B cells were cultured at 37°C in a 5% CO_2_ incubator. The cell culture medium was changed every 1-2 days, and the number cell morphology and number were observed with light microscope. When the number of cells reached 90%, they were subcultured at the ratio of 1 : 2. According to different experimental requirements, cells were cultured in high-glucose environment (glucose concentration: 30 mmol/L) and conventional environment (glucose concentration: 5.5 mmol/L).

### 2.2. Cell Scratch Assay

Experiment grouping was as follows. The hMSCs group normally cultured was taken as the control group, the group with 80 ummol/L CXCL-13 stimulant was taken as the CXCL-13 control group, the hMSCs cultured in high-glucose environment was taken as the cultured group in high-glucose environment, and the group cultured with 80 ummol/L CXCL-13 stimulant was taken as the stimulated group in high-glucose environment.

hMSCs were seeded in a 6-well plate at the density of 6 × 10^5^/well, and different reagents were added according to different conditions of each group. The cells were cultured in an incubator at constant temperature until 90% of cells were laid on the bottom of the plate. The bottom of plate was vertically scratched with 1 mL gun head. After 24 hours of the scratching, they were fixed with 4% paraformaldehyde solution for 60 minutes. The closure rate of the scratched area was calculated with ImageJ.

### 2.3. Transwell Chamber Assay

This essay aimed to investigate whether hMSCs migrate to human islet B cell culture medium containing CXCL-13 in high-glucose environment.

Grouping was as follows: human islet B cell group and human islet B cell + CXCL-13 group.

Immortalized hMSCs were cultured in Transwell chamber, and human islet B cells were cultured in a lower layer culture plate. According to groups, they were incubated in an incubator at constant temperature for 10 h without or with CXCL-13. The observation index was the number of migrated cells.

### 2.4. Western Blot

Experiment grouping was as follows: normal hMSCs group, normal human islet B cells group, normal hMSCs + human islet B cells group, high-glucose hMSCs group, high-glucose human islet B cells group, high-glucose hMSCs + human islet B cells group, high-glucose hMSCs + human islet B cells group, and hMSCs + B cells + AKT inhibitor group.

The protein of islet B cells was firstly extracted with lysis buffer, and the protein was quantitatively detected by BCA protein quantitative method. The extracted protein was placed in the refrigerator at −70°C. During the experiment, the protein sample was first added with 2x-volume buffer and then heated in boiling water for 20 minutes. Each electrophoresis channel was loaded with 30 ug, and the protein was transferred to PVDF membrane by electrophoresis. The 5% skimmed milk powder was sealed and shaken for 1 hour. Then, monoclonal antibodies against P53 and AKT were added, respectively. Horseradish peroxidase (HRP) labeled goat anti-rabbit IgG was added to make development and fixing with ECL kit. The internal reference was b-actin. Quantity One software was used to measure the integral optical density of each band after obtaining the target band.

### 2.5. RT-PCR

Experiment grouping: normal hMSCs group, normal human islet B cells group, normal hMSCs + human islet B cells group, high-glucose hMSCs group, high-glucose human islet B cells group, high-glucose hMSCs + human islet B cells group, high-glucose hMSCs + human islet B cells group, and hMSCs + B cells + AKT inhibitor group.

The islet B cells were inoculated on the 6-well plate at a density of 6 × 10^5^/well, and different reagents were added according to the culture conditions of each group for 48 h. After trypsin digestion, the RNA kit was used to extract the total RNA in the cells, and the mRNA was reverse-transcribed into cDNA with reverse transcription kit. Then, primers were designed according to the cDNA of rat Ki-67 gene to perform real-time PCR reactions. The relative expression level of Ki-67 was calculated using GADPH as internal reference.

### 2.6. Glucose Stimulated Insulin Secretion Experiment

Experiment grouping was as follows: normal human islet B cells group, normal hMSCs + human islet B cells group, high-glucose human islet B cells group, high-glucose hMSCs + human islet B cells group, high-glucose hMSCs + human islet B cells group, and hMSCs + B cells + AKT inhibitor group.

Human islet B cells were cultured according to the different culture conditions. After the cells grew to logarithmic phase, the cells were seeded into the 24-well plate. Different reagents were added according to the different culture conditions, and then the cells were cultured for 48 h. Insulin secretion was detected in the following ways: the cells were incubated with glucose-free Krebs–Ringer buffer for 30 min, and then the supernatant was discarded; 0.5 mL Krebs–Ringer buffer containing 3.3 mmol/L glucose was added to incubate the cells for 1 h, and the supernatant was collected; then, the cells were incubated with Krebs–Ringer buffer containing 16.7 mmol/L glucose for 1 h. The supernatant collected in two times was stored at −20°C. Insulin concentration was measured by radioimmunoassay.

### 2.7. Statistical Method

Statistical analysis of the data was performed with GraphPad Prism 8.0 software. Single factor square length analysis was used among multiple groups, and an independent sample *t*-test was used for comparison between two groups. The measurement data were expressed as mean ± standard deviation (*x* ± *s*), and *P* < 0.05 indicated that there was a statistical difference among all groups.

## 3. Result

### 3.1. CXCL-13 Can Promote the Migration of hMSCs in High-Glucose Environment

Transwell results showed that compared with the blank control group, the number of hMSCs migrated from Transwell chamber to the lower layer of culture medium was significantly increased (*P* < 0.05) when CXCL-13 was added to the lower layer of culture medium. After human islet B cells were cultured in the lower culture plate, it was found that the number of hMSCs transferred to the lower culture plate after adding CXCL-13 in the lower culture medium was still significantly higher than that in the group without CXCL-13 (*P* < 0.05) (Figure 1).

### 3.2. hMSCs Can Protect the Function of Islet B Cells in High-Glucose Environment

In order to demonstrate the effect of hMSCs on cell activity, CCK-8 assay showed that compared with that of normal medium, the activity of hMSCs and human islet B cells was significantly inhibited in high-glucose environment (*P* < 0.05). After the hMSCs were cocultured with human islet B cells, the cell activity was significantly higher than that of human islet B cells alone (*P* < 0.05). In order to investigate the effect of the hMSCs on islet B cell function in high-glucose environment, glucose stimulated insulin secretion experiment was performed. The results showed that compared with normal culture medium, the level of insulin secretion was significantly decreased (*P* < 0.05) under the stimulation of different concentrations of glucose in high-glucose environment. After the hMSCs were cocultured with human islet B cells, the level of insulin secretion was significantly higher than that of human islet B cells alone (*P* < 0.05). RT-PCR results showed that the expression of Ki-67 in hMSCs, and human islet B cells was significantly decreased in high-glucose culture environment (*P* < 0.05). WB test results showed that the expression of P53 in hMSCs and human islet B cells was significantly increased in high-glucose culture environment (*P* < 0.05). When hMSCs were cocultured with human islet B cells, the expression of Ki67 was significantly increased (*P* < 0.05), while the expression of P-53 was significantly decreased (*P* < 0.05) (Figure 2).

### 3.3. hMSCs Protect the Activity and Function of Islet B Cells through the AKT Signaling Pathway in High-Glucose Environment

In order to verify the specific molecular mechanism of the protective effect of hMSCs on the activity and function of islet B cells in high-glucose environment, islet B cells were cultured in high-glucose environment. CCK8 results showed that when AKT signaling pathway inhibitor was added, the cell activity was significantly inhibited (*P* < 0.05). The results of glucose stimulated insulin secretion experiment showed that with the addition of AKT inhibitor, insulin secretion of islet B cells was significantly inhibited (*P* < 0.05) by different concentrations of glucose. RT-PCR results showed that the expression of Ki-67 was significantly inhibited (*P* < 0.05) with the addition of AKT signaling pathway inhibitor. WB results showed that the expression of P53 was significantly increased and the expression of AKT was significantly decreased (*P* < 0.05) with the addition of ALT signaling pathway inhibitor (Figure 3).

## 4. Discussion

With the increasing number of diabetic patients, diabetes and its long-term complications have become a major threat to human health [5]. The prevalence of type 2 diabetes is significantly higher than that of type 1 diabetes, accounting for more than 90% of the total population of diabetes patients [1]. What is more, type 2 diabetes features insidious onset, and some patients are found islet dysfunction in clinical diagnosis, seriously affecting the recovery of patients. Therefore, it is difficult to develop a treatment method that can effectively protect the function of islets and delay the progress of this disease [17].

For the purpose of targeted treatment of type 2 diabetes, the specific mechanism of the occurrence and development of type 2 diabetes shall be firstly clarified. A high-glucose state can be found in diabetic patients, and long-term hyperglycemia will cause direct damage to islet B cells, promote the apoptosis of islet B cells, and inhibit their activity [4, 18]. Impaired islet B cell activity will further aggravate insulin resistance in patients and eventually lead to the reduction of insulin release and further improvement of blood glucose, forming a vicious circle [19]. Previous studies have shown that hyperglycemia could promote endoplasmic reticulum stress, oxidative stress, and inflammatory reaction in islet B cells and eventually lead to apoptosis [20]. This is similar to the result of this study. CCK8 results showed that, cultured in high-glucose environment, the activity of islet B cells was significantly decreased, the expression of cell proliferation-related protein (Ki-67) was significantly inhibited, and the expression of apoptosis related protein (P53) was significantly increased. Meanwhile, glucose stimulated insulin secretion experiment showed that insulin secretion stimulated by glucose was significantly decreased in high-glucose culture environment. These results effectively prove that in high-glucose environment, the activity and function of islet B cells can be significantly inhibited and their apoptosis can be promoted.

Patients with type 2 diabetes are in a pathological state, and the recovery of organ function will be quite limited under such conditions [7]. Previous treatments for type 2 diabetes showed no effect in restoring islet B cell function. On this basis, researchers try to restore the activity and function of damaged islet B cells with tissue engineering technology. Stem cells are expected to be used in the treatment of this disease due to their self-renewal and multidirectional differentiation abilities [6]. In order to verify the therapeutic effect of stem cells on type 2 diabetes, Bhansali [21] injected hMSCs in patients with type 2 diabetes through pancreatic artery puncture and found that the demand for insulin was significantly reduced after hMSCs injection. Previous studies have shown that the therapeutic effect of hMSCs can be realized by protecting the activity of islet B cells. Wu et al. [22] cocultured MSCs conditioned medium with islet cells and found that the expression of apoptosis related proteins of islet B cells in MSCs group decreased significantly, and the cell activity increased significantly. This was also verified in our study. In high-glucose culture environment, when hMSCs were cocultured with islet B cells, CCK8 results showed that the cell activity was significantly increased, the expression of proliferation-related protein Ki-67 was significantly increased, and the expression of apoptosis related protein P53 was significantly decreased. The results of glucose stimulated insulin secretion experiment showed that the amount of insulin secretion was significantly increased. These results indicated that hMSCs can effectively protect the activity of islet B cells and inhibit their apoptosis in high-glucose environment.

Previous studies have shown that directional induction of MSCs to the injured area is more conducive to achieve self-renewal [23]. Previous studies have shown that CXCL-13, a subfamily of CXC in chemokine family, could bind to CXCR5 receptor on the surface of MSCs, thus promoting the migration of MSCs [24]. Shen et al. [25] found that the migration and movement of hMSCs were significantly improved after CXCL-13 was applied to hMSCs. Qian et al. [26] found that the migration of hMSCs was significantly improved after Bushen Huoxue Decoction was applied to hMSCs, and the expression of CXCL-13 was also significantly increased. Correlation analysis showed that the migration ability of hMSCs was positively correlated with the expression of CXCL-13. These results showed that CXCL-13 could effectively promote the migration and movement of hMSCs.

AKT signaling pathway, a cascade signaling pathway for intracellular information transmission, plays a regulatory and guiding role in cell proliferation, differentiation, apoptosis, and other cellular behaviors [27]. Its specific mechanism in cells is that AKT induces cells to enter S phase from resting state by activating cyclins to promote cell proliferation [19]. AKT can also control the expression of cyclin inhibitors, thus further regulating the proliferation and differentiation of cells [28]. At the same time, AKT signaling pathway can regulate the expression of P53 in cells. As a proliferation suppressor protein, P53 can effectively promote cell cycle arrest, cell apoptosis, and other events. Previous studies have shown that P53 is closely related to the proliferation and migration of various cells [29]. In order to study the specific mechanism of hMSCs protecting the activity of islet B cells, hMSCs were cocultured with islet B cells in high-glucose culture environment. The results showed that the expression of AKT was significantly upregulated. In order to further verify the specific role of AKT, AKT specific inhibitor LY294002 was added to the cocultured group of hMSCs and islet B cells. When AKT signaling pathway was blocked, CCK8 results showed that cell activity was significantly inhibited, the expression of proliferation related protein Ki-67 was inhibited, and the expression of apoptosis related protein P53 was significantly upregulated. These results indicated that the protective effect of hMSCs on islet B cells was significantly inhibited with the addition of LY294002 and further proved that hMSCs could protect the activity of islet B cells through AKT signaling pathway in high-glucose environment.

## 5. Conclusion

AKT signaling pathway plays an important role to realize the protective effect of hMSCs on the function of islet B cells in high-glucose environment. It can be concluded from the above results that hMSCs play a protective role on islet B cells by activating AKT signaling pathway in high-glucose culture, promoting the proliferation of islet B cells and inhibiting the apoptosis of islet B cells.

However, stem cell therapy still has some defects and limitations. First of all, it still requires great efforts to explore the way to effectively migrate stem cells to damaged tissues and play their role [10]. Secondly, the specific mechanism of hMSCs in the treatment of islet B cell injury in high-glucose environment is not clear. What is more, no study has reported if CXCL-13 can promote the migration of hMSCs to islet B cells in high-glucose environment. The results of scratch test showed that CXCL-13 could significantly promote the migration and motility of hMSCs in high-glucose culture environment. Transwell experiment showed that CXCL-13 could effectively induce hMSCs to migrate to islet B cells in high-glucose culture environment. These results indicated that CXCL-13 can be used as an effective inducer to promote the migration of hMSCs to damaged islet B cells in high-glucose culture environment.

In conclusion, CXCL-13 can effectively promote the migration and movement of hMSCs to islet B cells in high-glucose environment. At the same time, hMSCs can protect islet B cells from high-glucose damage through AKT signaling pathway and maintain insulin secretion function of islet B cells. The results also provide a reliable theoretical basis for the treatment of type 2 diabetes with hMSCs.

## Figures and Tables

**Figure 1:** Effect of CXCL-13 on the migration of hMSCs in high-glucose environment. Note: transwell experiment showed that CXCL-13 could promote the migration of hMSCs in high-glucose environment (*P* < 0.05) and also promote the migration of hMSCs to islet B cells (*P* < 0.05).

**Figure 2:** Effect of hMSCs on islet B cells in high-glucose environment. (a) CCK8 assay showed that the cell activity in high-glucose culture environment was significantly lower than that in normal culture environment. In the high-glucose culture environment, when the hMSCs were cocultured with B cells, the cell activity was significantly higher than that of human islet B cells alone (*P* < 0.05). (b) The results of glucose stimulated insulin secretion experiment showed that the ability of insulin secretion of islet B cells was significantly decreased in high-glucose culture environment, and when the hMSCs were cocultured with B cells, the ability of insulin secretion of islet B cells was significantly increased (*P* < 0.05). (c) The expression of P53 was detected by WB assay. (d) RT-PCR analysis showed that the expression of Ki67 was significantly decreased in high-glucose culture environment, and when the hMSCs were cocultured with B cells, the expression of Ki67 was significantly increased (*P* < 0.05) compared with that of B cells alone in high-glucose culture environment. (e) WB results showed that the expression of P53 was significantly increased in high-glucose culture environment compared with that in normal culture environment, and when the hMSCs were cocultured with B cells, the expression of P53 was significantly decreased (*P* < 0.05) compared with that of B cells alone in high-glucose culture environment.

**Figure 3:** hMSCs protect the activity and function of islet B cells through the AKT signaling pathway in high-glucose environment. (a) CCK8 assay showed that the cell activity was significantly inhibited (*P* < 0.05) when AKT signaling pathway was inhibited. (b) The results of glucose stimulated insulin secretion experiment showed that when AKT signaling pathway was inhibited, the insulin secretion of islet B cells was significantly decreased (*P* < 0.05). (c) The expression of AKT was detected by WB assay. (d) The expressions of AKT and P53 in islet B cells of different groups were detected by WB assay. (e) WB results showed that the expression of AKT in islet B cells was significantly increased in high-glucose culture environment, and the expression of AKT was significantly increased (*P* < 0.05) when hMSCs were added into islet B cells in high-glucose culture environment compared with that in normal high-glucose culture environment. (f) The expression of Ki-67 was detected by RT-PCR. The results showed that the expression of Ki-67 was also significantly inhibited (*P* < 0.05) with the addition of AKT signaling pathway inhibitor. (g) WB results showed that the expression of P53 was significantly increased (*P* < 0.05) with the addition of AKT signaling pathway inhibitor. (h) WB results showed that the expression of AKT was significantly inhibited (*P* < 0.05) with the addition of AKT signaling pathway inhibitor.

## Data Availability

The datasets used and/or analyzed during the present study are available from the corresponding author on reasonable request.
